The article "1,25‐Dihydroxyvitamin D exerts an antiaging role by activation of Nrf2‐antioxidant signaling and inactivation of p16/p53‐senescence signaling" was retracted in 2024. Reasons: manipulated images; errors in the images; duplicated images; unreliable data.

# 1,25‐Dihydroxyvitamin D exerts an antiaging role by activation of Nrf2‐antioxidant signaling and inactivation of p16/p53‐senescence signaling

**DOI:** 10.1111/acel.12951

**Published:** 2019-03-24

**Authors:** Lulu Chen, Renlei Yang, Wanxin Qiao, Wei Zhang, Jie Chen, Li Mao, David Goltzman, Dengshun Miao

**Affiliations:** ^1^ State Key Laboratory of Reproductive Medicine, The Research Center for Bone and Stem Cells, Department of Anatomy, Histology and Embryology Nanjing Medical University Nanjing China; ^2^ Department of Endocrinology, Huai'an First People's Hospital Nanjing Medical University Huai'an China; ^3^ Calcium Research Laboratory, McGill University Health Centre and Department of Medicine McGill University Montreal Quebec Canada

**Keywords:** aging, cell senescence, Nrf2, p16 and p53, vitamin D

## Abstract

We tested the hypothesis that 1,25‐dihydroxyvitamin D_3_[1α,25(OH)_2_D_3_] has antiaging effects via upregulating nuclear factor (erythroid‐derived 2)‐like 2 (Nrf2), reducing reactive oxygen species (ROS), decreasing DNA damage, reducing p16/Rb and p53/p21 signaling, increasing cell proliferation, and reducing cellular senescence and the senescence‐associated secretory phenotype (SASP). We demonstrated that 1,25(OH)_2_D_3_‐deficient [1α(OH)ase^−/−^] mice survived on average for only 3 months. Increased tissue oxidative stress and DNA damage, downregulated Bmi1 and upregulated p16, p53 and p21 expression levels, reduced cell proliferation, and induced cell senescence and the senescence‐associated secretory phenotype (SASP) were observed. Supplementation of 1α(OH)ase^−/−^ mice with dietary calcium and phosphate, which normalized serum calcium and phosphorus, prolonged their average lifespan to more than 8 months with reduced oxidative stress and cellular senescence and SASP. However, supplementation with exogenous 1,25(OH)_2_D_3_ or with combined calcium/phosphate and the antioxidant *N*‐acetyl‐l‐cysteine prolonged their average lifespan to more than 16 months and nearly 14 months, respectively, largely rescuing the aging phenotypes. We demonstrated that 1,25(OH)_2_D_3_exerted an antioxidant role by transcriptional regulation of Nrf2 via the vitamin D receptor (VDR). Homozygous ablation of p16 or heterozygous ablation of p53 prolonged the average lifespan of 1α(OH)ase^−/−^ mice on the normal diet from 3 to 6 months by enhancing cell proliferative ability and reducing cell senescence or apoptosis. This study suggests that 1,25(OH)_2_D_3_ plays a role in delaying aging by upregulating Nrf2, inhibiting oxidative stress and DNA damage，inactivating p53‐p21 and p16‐Rb signaling pathways, and inhibiting cell senescence and SASP.

## 1 INTRODUCTION

The active form of vitamin D, 1,25 dihydroxyvitamin D_3_ [1,25(OH)_2_D_3_], generated by the 25‐hydroxyvitamin D 1α‐hydroxylase [1α(OH)ase] enzyme is known to bind to its cognate receptor, the vitamin D receptor (VDR) (Li et al., 1997) and to increase intestinal calcium and phosphorus absorption and enhance renal calcium reabsorption (Fleet, 2017). These ions may be involved in a number of critical physiologic regulatory functions. However, there is increasing evidence that vitamin D may also play an important role in the process of aging. Epidemiological surveys have shown that vitamin D deficiency is associated with high mortality (Zittermann, Gummert, & Borgermann, 2009) and vitamin D deficient women have shortened telomere length and relatively short lifespan (Richards et al., 2007). Furthermore, VDR mice deficient in the gene encoding the vitamin D receptor (*Vdr*) (VDR knockout [KO] mice) also exhibit aging phenotypes (Haussler et al., 2010; Keisala et al., 2009) and 1,25(OH)_2_D_3_ can increase levels of the protein Klotho that has enzyme/coreceptor properties and that protects against aging phenotypes such as skin atrophy, osteopenia, and atherosclerosis (Haussler et al., 2016). VDR KO mice and mice with targeted deletion of *Cyp27b1*which encodes the 1α(OH)ase enzyme [1α(OH)ase^−/−^ mice] have been compared. Although they share many phenotypical changes including premature aging, nevertheless, p53 levels are lower in VDR knockout mice than in wild‐type while higher in *Cyp27b1* knockouts (Keisala et al., 2009). Whether this indicates that VDR or 1,25(OH)_2_D_3_ exerts independent mechanistic effects in this regard remains to be determined. It has also been suggested that vitamin D deficiency could also contribute to the initiation of age‐related diseases such as Alzheimer's disease, Parkinson's disease, multiple sclerosis (Mokry et al., 2016), hypertension, and cardiovascular disease (Berridge, 2015a). Many of these diseases are often associated with alterations in both calcium and redox signaling, both of which may be regulated by 1,25(OH)_2_D_3_ operating together with Klotho and nuclear factor (erythroid‐derived 2)‐like 2 (Nrf2), the basic leucine zipper (bZIP) protein that regulates the expression of antioxidant proteins that protect against oxidative damage triggered by injury and inflammation (Berridge, 2015a,2015b; Moi, Chan, Asunis, Cao, & Kan, 1994). Interestingly, hypervitaminosis D, at least as seen in FGF‐23‐ and klotho‐deficient mice, also leads to premature aging. Whether this indicates the presence of a “U‐shaped curve” for the effects of 1,25(OH)_2_D_3_ on aging or whether the aging effects of Klotho and FGF23 deficiency in these models supersedes the effects of the high 1,25(OH)_2_D_3_ is unclear. There is therefore reason to suspect that reductions in the rate of aging and the onset of these diseases could be achieved by maintaining normal 1,25(OH)_2_D_3_ levels and thereby preventing the dysregulation of the calcium and redox signaling pathways. However, although vitamin D appears to play an important role in the aging process, the mechanisms of vitamin D deficiency leading to aging require further study.

The article "1,25‐Dihydroxyvitamin D exerts an antiaging role by activation of Nrf2‐antioxidant signaling and inactivation of p16/p53‐senescence signaling" was retracted in 2024. Reasons: manipulated images; errors in the images; duplicated images; unreliable data.

Increasing oxidative stress, a major characteristic of aging, has been implicated in a variety of age‐related pathologies. In aging, oxidant production from several sources is increased, whereas antioxidant enzymes, the primary lines of defense, are decreased (Zhang, Davies, & Forman, 2015).The close link between oxidative stress and aging is evident in mice with genetic ablation of the redox‐sensitive transcription factor Nrf2 (Nrf2 knockout mice), which display some phenotypes of aging that results from a decline in antioxidative pathways (Cheung et al., 2014; Hayes & Dinkova‐Kostova, 2014). A recent report showed that upregulation of the Nrf2 pathway rescued many of the cellular phenotypes of progeria (Kubben et al., 2016). Nrf2 protects organisms against detrimental effects of reactive oxygen species (ROS) through activation of an array of antioxidative and detoxification response genes (Kubben et al., 2016). Previous in vivo studies have demonstrated that vitamin D is a very effective antioxidant, with a capacity to inhibit zinc‐induced oxidative stress in the central nervous system that is 10^3^ times greater than vitamin E analogues (Lin, Chen, & Chao, 2005). Vitamin D has also been reported to be as potent as vitamin E in increasing the activities of erythrocyte superoxide dismutase (SOD) and catalase in atopic dermatitis patients (Javanbakht, 2010). However, whether this antioxidant effect of vitamin D contributes to its antiaging action is unclear.

Reactive oxygen species can induce DNA damage and activate a DNA damage response, subsequently leading to activation of p53 (Rai et al., 2009). p53 functions as a transcription factor involved in cell‐cycle control, DNA repair, apoptosis, and cellular stress responses. However, in addition to inducing cell growth arrest and apoptosis, p53 activation also modulates cellular senescence and organismal aging (Rufini, Tucci, Celardo, & Melino, 2013). p16^INK4a^, a cyclin‐dependent kinase inhibitor, tumor suppressor, and biomarker of aging, is another major mediator for cellular senescence. The gradual accumulation of p16 expression during physiological aging and several aging‐associated diseases directly implicates this well‐established effector of senescence in the aging process (Krishnamurthy et al., 2004). Senescent cells have been proposed as a target for interventions to delay the aging process and its related diseases or to improve disease treatment. Therapeutic interventions geared toward senescent cells might allow reduction in diseases of aging and improvement of health. Baker and colleagues found that the elimination of p16^Ink4a^‐expressing cells increased lifespan and ameliorated a range of age‐dependent, disease‐related abnormalities, including kidney dysfunction and abnormalities in heart and fat tissue (Baker et al., 2016,2011). Previous studies have suggested that adequate levels of vitamin D may also be beneficial in maintaining DNA integrity. The potential for vitamin D to reduce oxidative damage to DNA in humans has been suggested by clinical trials where vitamin D supplementation reduced 8‐hydroxy‐2′‐deoxyguanosine, a marker of oxidative damage, in colorectal epithelial crypt cells (Smith et al., 1999) and in human lymphocytes, and pulmonary carcinoma cells (Halicka et al., 2012). However, whether 1,25(OH)_2_D_3_ can employ any of the above mechanisms to help prevent aging is unclear.

The article "1,25‐Dihydroxyvitamin D exerts an antiaging role by activation of Nrf2‐antioxidant signaling and inactivation of p16/p53‐senescence signaling" was retracted in 2024. Reasons: manipulated images; errors in the images; duplicated images; unreliable data.

In the present studies, we therefore tested the hypothesis that 1α,25(OH)_2_D_3_ has antiaging effects via upregulating Nrf2, reducing ROS, decreasing DNA damage, reducing p16/Rb and p53/p21 signaling, increasing cell proliferation, and reducing cellular senescence and the senescence‐associated secretory phenotype (SASP). We addressed the characteristics of the aging phenotype and of 1,25(OH)_2_D_3_‐related mechanisms involved, using 1α(OH)ase^−/−^ mice; using mice with homozygous deletion of both 1α(OH)ase and p16 genes [1α(OH)ase^−/−^p16^−/−^ mice]; and using mice with homozygous deletion of the 1α(OH)ase and heterozygous deletion of the p53 gene [1α(OH)ase^−/−^p53^+/−^ mice].

## 2 RESULTS

### 2.1 1,25(OH)_2_D_3_deficiency accelerates organismal aging

Serum levels of calcium and phosphorus levels were significantly decreased, 1,25(OH)_2_D_3_ levels were undetectable, and 25(OH)D and parathyroid hormone (PTH) levels were significantly increased (Figure 1a–e); body size (Supporting Information Figure S1) and body weight (Figure 1g) were reduced in 10‐week‐old 1α(OH)ase^−/−^ mice on a normal diet compared with their wild‐type littermates. The average lifespan of 1α(OH)ase^−/−^ mice on a normal diet was 91 days (67–120 days; Figure 1f). Aging phenotypes were detected in multiple organs from these 1α(OH)ase^−/−^ mice. The skin was thinner (Figure 1h,i), and collagen deposition in skin was reduced (Figure 1j,k). Levels of ROS were increased significantly in the skin, liver, and kidney (Figure 2a–c and Supporting Information Figure S3), whereas cells immunopositive for the antioxidant enzyme, SOD2 (Figure 2d,e and Supporting Information Figure S2a,b), and PrdxI protein expression levels in the skin and liver (Figure 2h,i, and Supporting Information Figure 2e,f) were decreased dramatically in 1α(OH)ase^−/−^ mice. Cells in the skin and kidney positive for the DNA damage marker, phosphorylation of histone protein H2AX (γ‐H2AX) were increased significantly in 1α(OH)ase^−/−^ mice (Figure 2f,g and Supporting Information Figure S2c,d). Protein expression levels of the oncogene Bmi1 were downregulated dramatically in the skin and liver (Figure 2j,k and Supporting Information Figure S2g,h), whereas protein expression levels of tumor suppressor genes including p16, p53, and p21 were upregulated significantly in the skin and liver of 1α(OH)ase^−/−^ mice (Figure 2j,k and Supporting Information Figure S2i–n). The percentage of Ki67‐positive cells in the skin, liver, and kidney were clearly reduced (Figure 3a,b and Supporting Information Figure S3a–d), whereas senescence‐associated β‐galactosidase (SA‐β‐gal)‐positive areas in the skin, kidney, and lung (Figure 3c–f and Supporting Information Figure S4c–f) and senescence‐associated secretory phenotype (SASP) molecules including TNFα, IL‐1α and β, IL‐6, Mmp 3 and 13 were increased significantly in the skin, kidney, liver, and lung (Figure 3g,h and Supporting Information Figure S3g,h) of 1α(OH)ase^−/−^ mice. These results demonstrated that 1,25(OH)_2_D_3_deficiency accelerated organismal aging by inhibiting cell proliferation and inducing cell senescence and SASP via increased oxidative stress, DNA damage, and activation of p16 and p53 signaling pathways.

The article "1,25‐Dihydroxyvitamin D exerts an antiaging role by activation of Nrf2‐antioxidant signaling and inactivation of p16/p53‐senescence signaling" was retracted in 2024. Reasons: manipulated images; errors in the images; duplicated images; unreliable data.

**Figure 1:** The effects of a high calcium/phosphate diet, of 1,25(OH)_2_D_3,_ and of antioxidant supplementation on lifespan, body weight, and skin morphology in 1α(OH)ase^−/−^ mice. After weaning, sex‐matched wild‐type (WT) and 1α(OH)ase^−/−^ (KO) mice were fed a normal diet (ND) or a “rescue diet” diet (RD) or received thrice weekly subcutaneous injections of vehicle (ND) or 1,25(OH)_2_D_3_ (1 μg/kg) (VD), or were fed a rescue diet with 1 mg/ml NAC in drinking water (RD + NAC). (a) Serum calcium, (b) phosphorus, (c) 1,25(OH)_2_D_3_, (d) 25(OH)D, and (e) PTH. (f) Survival rate of the mice; (g) body weight. Representative micrographs of skin sections stained (h) with H&E or (j) histochemically for total collagen (T‐Col). Scale bars represent 200 μm in c and e. (i) Skin thickness and (k) total collagen‐positive area (%). Each value is the mean ± *SEM* of determinations in five mice of each group. *p < 0.05; **p < 0.01; ***p < 0.001 compared with WT mice. ^#^ *p < *0.05; ^##^ *p < *0.01 compared with ND KO mice. ^&^ *p < *0.05; ^&&^ *p < *0.01 compared with RD KO mice

**Figure 2:** The effects of a high calcium/phosphate diet, of 1,25(OH)_2_D_3,_ and of antioxidant supplementation on oxidative stress, DNA damage, and protein expression of oncogenes and tumor suppressive genes in 1α(OH)ase^−/−^ mice. Mice from each group were treated as described in Figure 1. ROS levels in freshly isolated cells of (a) skin, (b) liver, and (c) kidney from 10‐week‐old wild‐type (WT) and 1α(OH)ase^−/−^ (KO) mice. Representative micrographs of skin sections stained immunohistochemically for (d) SOD2 and (f) γ‐H2AX. Scale bars represent 50 μm in d and f. (e) The percentage of SOD2‐positive cells of skin and (g) the percentage of γ‐H2AX‐positive cells of skin; (h) representative Western blots of skin extracts to determine Prdx I protein levels. β‐actin was used as loading control. (i) Skin Prdx I and Bmi1, p16, p53 and p21 protein levels in (j) skin and (k) liver relative to β‐actin protein levels were assessed by densitometric analysis and expressed as a percentage of the levels of vehicle‐treated wild‐type mice fed the normal diet (ND).Each value is the mean ± *SEM* of determinations in five mice of each group. *p < 0.05; **p < 0.01; ***p < 0.001 compared with WT mice. ^#^ *p < *0.05; ^##^ *p < *0.01 compared with ND KO mice. ^&^ *p < *0.05; ^&&^ *p < *0.01 compared with RD KO mice

**Figure 3:** The effects of a high calcium/phosphate diet, of 1,25(OH)_2_D_3,_ and of antioxidant supplementation on cell proliferation and senescence in 1α(OH)ase^−/−^ mice. Mice from each group were treated as described in Figure 1. (a) Representative micrographs of paraffin sections from 10‐week‐old wild‐type (WT) and 1α(OH)ase^−/−^ (KO) mice stained immunohistochemically for ki67 in skin (b) The percentage of ki67‐positive cell number relative to total cell number in skin. Representative micrographs of sections from 10‐week‐old WT and KO mice stained histochemically for senescence‐associated β‐galactosidase (SA‐β‐gal) in (c) skin and (e) kidney. Scale bars represent 50 μm in a, c, and e. The percentage of SA‐β‐gal‐positive area in (d) skin and (f) kidney. RT–PCR of (g) skin, and (h) kidney tissue extracts for expression of TNFα, IL‐1α and β, IL‐6, Mmp 3 and 13. Messenger RNA expression assessed by real‐time RT–PCR is calculated as a ratio relative to GAPDH, and expressed relative to ND WT mice. Each value is the mean ± *SEM* of determinations in five mice of each group. *p < 0.05; **p < 0.01; ***p < 0.001 compared with WT mice. ^#^ *p < *0.05; ^##^ *p < *0.01; ^###^ *p < *0.001 compared with ND KO mice. ^&^ *p < *0.05; ^&&^ *p < *0.01; ^&&&^ *p < *0.001 compared with RD KO mice

The article "1,25‐Dihydroxyvitamin D exerts an antiaging role by activation of Nrf2‐antioxidant signaling and inactivation of p16/p53‐senescence signaling" was retracted in 2024. Reasons: manipulated images; errors in the images; duplicated images; unreliable data.

### 2.2 Supplementation with calcium and phosphate or with exogenous 1,25(OH)_2_D_3_postpones aging induced by 1,25(OH)_2_D_3_deficiency

To determine whether 1,25(OH)_2_D_3_deficiency‐induced aging is calcium‐/phosphorus‐dependent or 1,25(OH)_2_D_3_‐dependent, 1α(OH)ase^−/−^ mice and their wild‐type littermates were fed a high calcium/phosphate (rescue) diet after weaning to normalize their serum calcium and phosphorus levels (Panda et al., 2004), or were injected with 1,25(OH)_2_D_3_subcutaneously. Their phenotypes were compared with genotype‐matched mice on the normal diet. Results revealed that, in 1α(OH)ase^−/−^ mice, the average lifespan was prolonged to 252 days (154–465 days) in 1α(OH)ase^−/−^ mice on the rescue diet, and to 487 days (358–540 days) in 1α(OH)ase^−/−^ mice with exogenous 1,25(OH)_2_D_3_ supplementation (Figure 1f). Serum 1,25(OH)_2_D_3_was undetectable in 1α(OH)ase^−/−^ mice on the rescue diet, but reached near normal levels in 1α(OH)ase^−/−^ mice with exogenous 1,25(OH)_2_D_3_ supplementation (Supporting Information Figure S1c). Serum calcium, phosphorus, and PTH levels were normalized in 1α(OH)ase^−/−^ mice supplemented with either dietary calcium/phosphate or exogenous 1,25(OH)_2_D_3_injection (Figure 1a,b,e), whereas serum 25(OH)D levels were increased in 1α(OH)ase^−/−^ mice on the rescue diet and reduced in 1α(OH)ase^−/−^ mice with exogenous 1,25(OH)_2_D_3_injection (Figure 1d). Body size (Supporting Information Figure S1) and body weight (Figure 1g) were increased in 1α(OH)ase^−/−^ mice on the rescue diet and were near normal in 1α(OH)ase^−/−^ mice with exogenous 1,25(OH)_2_D_3_ supplementation. The thickness of skin and collagen deposition in skin were increased in 1α(OH)ase^−/−^ mice on the rescue diet, but increased more dramatically in 1α(OH)ase^−/−^ mice with exogenous 1,25(OH)_2_D_3_ supplementation (Figure 1h–k). ROS levels (Figure 2a–c, Supporting Information Figure S3) and γ‐H2AX‐positive cells in the skin and kidney (Figure 2f,g and Supporting Information Figure S2c,d) were reduced significantly in 1α(OH)ase^−/−^ mice on the rescue diet but reduced more markedly by exogenous 1,25(OH)_2_D_3_ supplementation. In contrast, SOD2 immunopositive cells in skin and liver (Figure 2d,e, Supporting Information Figure S2a,b) were increased significantly by the rescue diet in 1α(OH)ase^−/−^ mice and more markedly increased by exogenous 1,25(OH)_2_D_3_ supplementation. Peroxiredoxin (Prdx) I protein expression levels in the skin and liver (Figure 2h,i and Supporting Information Figure S2e,f), and Bmi1, p16, p53, and p21 protein expression levels in the skin and liver were not altered significantly in 1α(OH)ase^−/−^ mice on the rescue diet, but were normalized in 1α(OH)ase^−/−^ mice with exogenous 1,25(OH)_2_D_3_ supplementation (Figure 2j,k and Supporting Information Figure S2g–n). The percentage of Ki67‐positive cells in the skin, liver, and kidney (Figure 3a,b and Supporting Information Figure S3a–d) were not altered in 1α(OH)ase^−/−^ mice on the rescue diet relative to those on the normal diet, but the percentage of Ki67‐positive cells was increased in 1α(OH)ase^−/−^ mice with exogenous 1,25(OH)_2_D_3_ supplementation. SA‐β‐gal‐positive areas in the skin, kidney, and lung (Figure 3c–f and Supporting Information Figure S4c–f) and SASP molecules including TNFα, IL‐1α and β, IL‐6, Mmp 3 and 13 in the skin, kidney, liver, and lung (Figure 3g,h and Supporting Information Figure S4g,h) were reduced significantly in 1α(OH)ase^−/−^ mice on the rescue diet but more extensively by exogenous 1,25(OH)_2_D_3_supplementation. These results demonstrate that the supplementation of calcium and phosphate could prolong the lifespan of 1,25(OH)_2_D_3_‐deficient mice in association with inhibiting oxidative stress, DNA damage, cell senescence, and SASP, whereas supplementation with exogenous 1,25(OH)_2_D_3_ could more dramatically postpone aging induced by 1,25(OH)_2_D_3_ deficiency by inhibiting oxidative stress, DNA damage, and p16 and p53 signaling pathways, subsequently stimulating cell proliferation and inhibiting cell senescence and SASP.

The article "1,25‐Dihydroxyvitamin D exerts an antiaging role by activation of Nrf2‐antioxidant signaling and inactivation of p16/p53‐senescence signaling" was retracted in 2024. Reasons: manipulated images; errors in the images; duplicated images; unreliable data.

### 2.3 Supplementation of antioxidant NAC postpones aging induced by 1,25(OH)_2_D_3_ deficiency

To further determine whether the action of 1,25(OH)_2_D_3_on delaying aging is mediated by its antioxidative role, 1α(OH)ase^−/−^ mice and their wild‐type littermates on the rescue diet were supplemented with the antioxidant NAC in drinking water. Serum 1,25(OH)_2_D_3_ was undetectable, and serum calcium, phosphorus, and PTH levels were normalized, whereas serum 25(OH)_2_D levels were increased in 1α(OH)ase^−/−^ mice on the rescue diet supplemented with NAC (Supporting Information Figure S1a–e). Their aging phenotypes were then compared with genotype‐matched mice on the rescue diet alone or on a normal diet supplemented with exogenous 1,25(OH)_2_D_3_. We found that with NAC supplementation in 1α(OH)ase^−/−^ mice on the rescue diet, the average lifespan was prolonged to 409 days (320–540 day) which was 157 days longer than those on the rescue diet alone, but was 78 days shorter than with exogenous 1,25(OH)_2_D_3_ supplementation (Figure 1f). Body size (Supporting Information Figure S1) and body weight (Figure 1b) were not further increased in 1α(OH)ase^−/−^ mice on the rescue diet with NAC supplementation compared with these on the rescue diet alone. The thickness of skin and collagen deposition in skin were increased significantly in 1α(OH)ase^−/−^ mice on the rescue diet with NAC supplementation compared with these on the rescue diet alone, and levels were comparable to those seen with exogenous 1,25(OH)_2_D_3_ supplementation (Figure 1h–k). Alterations in ROS levels (Figure 2a–c and Supporting Information Figure S3), SOD2 immunopositive cells (Figure 2d,e, and Supporting Information Figure 2a,b), and Prdx I protein expression levels in the skin and liver (Figure 2h,i and Supporting Information Figure S2e,f), γ‐H2AX‐positive cells in the skin and kidney (Figure 2f,g and Supporting Information Figure S2c,d), Bmi1, p16, p53, and p21 protein expression levels in the skin and liver (Figure 2j,k and Supporting Information Figure S2g–n), the percentage of Ki67 positive cells in the skin, liver, and kidney (Figure 3a,b and Supporting Information Figure S4a–d), SA‐β‐gal‐positive areas in the skin, kidney, and lung (Figure 3c–f and Supporting Information Figure S3e,f), SASP molecules including TNFα, IL‐1α and β, IL‐6, Mmp 3 and 13 in the skin, kidney, liver, and lung (Figure 3g,h and Supporting Information Figure 4g,h) were all significantly reversed in 1α(OH)ase^−/−^ mice on the rescue diet with NAC supplementation compared with these on the rescue diet alone, and levels were comparable to those seen with exogenous 1,25(OH)_2_D_3_supplementation. These results demonstrated that the antiaging effects of combined calcium/phosphate and antioxidative NAC supplementation were almost as efficacious as the effects observed with exogenous 1,25(OH)_2_D_3_supplementation.

The article "1,25‐Dihydroxyvitamin D exerts an antiaging role by activation of Nrf2‐antioxidant signaling and inactivation of p16/p53‐senescence signaling" was retracted in 2024. Reasons: manipulated images; errors in the images; duplicated images; unreliable data.

**Figure 4:** 1,25(OH)_2_D_3_ exerts an antioxidant role by transcriptional regulation of Nrf2 mediated through the vitamin D receptor. MEFs from wild‐type and VDR knockout (VDR KO) mice were treated with 10^−9^–10^−7^ M 1,25(OH)_2_D_3_ for 24 hr, and the mRNA relative expression levels of Nrf2 in MEFs were examined by real‐time RT–PCR. *p < 0.05; **p < 0.01; ***p < 0.001 compared with control cultures. (b) VDR‐like elements in mouse Nrf2 promoter region and the mutated VDRE sequence highlighted in red color (upper panels); structure schematic diagram of pGL3‐Nrf2 promoter reporter plasmid and mutant pGL3‐Nrf2 promoter reporter plasmid. (c) Luciferase activity driven by Nrf2 promoter, more dramatically by 1,25(OH)_2_D_3_treatment_,_but not driven by Nrf2 luciferase reporter with mutated VDRE treated without/with 1,25(OH)_2_D_3_. **p < 0.01; ***p < 0.001 compared with negative control. ^###^ *p < *0.001 compared with genotype‐matched cells. (d) Nrf2 promoter sequences could be recovered by PCR from VDR immunoprecipitates but not from pre‐immune IgG immunoprecipitates. (e) The mRNA level of Nrf2 in Vector (SiControl) or SiNrf2 transfected MEFs. ***p < 0.001 compared with SiControl. (f–i) Messenger RNA expression assessed by real‐time RT–PCR is calculated in Vector (real‐time RT–PCR is calculated in Vector (Si‐Control) or siNrf2 transfected MEFs as a ratio relative to GAPDH, and expressed relative to SiControl MEFs. Each value is the mean ± *SEM* of determinations in triplicated cultures. *p < 0.05; ***p < 0.001 compared with wild‐type MEFs. ^#^ *p < *0.05; ^###^ *p* < 0.001 compared with SiControl. ^&^ *p < *0.05; ^&&&^ *p < *0.001 compared with SiNrf2

The article "1,25‐Dihydroxyvitamin D exerts an antiaging role by activation of Nrf2‐antioxidant signaling and inactivation of p16/p53‐senescence signaling" was retracted in 2024. Reasons: manipulated images; errors in the images; duplicated images; unreliable data.

### 2.4 1,25(OH)_2_D_3_ exerts an antioxidant role by transcriptional regulation of Nrf2 mediated through the VDR

In view of the fact that the transcription factor Nrf2 is a master regulator of antioxidants, mouse embryonic fibroblasts (MEFs) from wild‐type and VDR knockout (VDR KO) mice were treated with 10^−9^–10^−7^ M 1,25(OH)_2_D_3_ for 24 hr, and the mRNA expression levels of Nrf2 in MEFs were examined by real‐time RT–PCR. We found that the expression levels of Nrf2 were upregulated significantly in 1,25(OH)_2_D_3_‐treated MEFs from wild‐type mice in a dose‐dependent manner, but not in these from VDR KO mice (Figure 4a). To confirm that 1,25(OH)_2_D_3_ regulates Nrf2 via the VDR at a transcriptional level, a VDRE‐like sequence in the 5′‐flanking regions of the Nrf2 promoter, sequence NT039207 (retrieved from the NCBI mouse genome database), was identified by computer‐aided analysis at position −460 (Figure 4b). Using mouse genomic DNA as a template, PCR was used to amplify the whole promoter segment −613 to −361. The PCR products without and with mutated VDRE (Figure 4b) were then cloned into pGL3‐basic vectors (Nrf2‐PGL3, Nrf2‐PGL3 mutant), which were transiently transfected into MEFs. Luciferase activities were increased significantly in MEFs transfected with Nrf2‐PGL3 plasmid compared with the empty plasmid and were increased more dramatically in 1,25(OH)_2_D_3_‐treated MEFs transfected with Nrf2‐PGL3 plasmid. In contrast, luciferase activities were not increased in MEFs transfected with Nrf2‐PGL3 mutant plasmid compared with the empty plasmid, and 1,25(OH)_2_D_3_ failed to activate this mutant reporter (Figure 4c). These results confirmed that the promoter region containing the predicted VDR binding sites of the Nrf2 gene is sufficient to promote transcription and supported the hypothesis that Nrf2 transcriptional activation could be mediated by the VDR. We next assessed whether the VDR has the ability to physically bind the Nrf2 promoter using a chromatin immunoprecipitation (ChIP) approach. The Nrf2 promoter sequence was amplified in the total input sample as a positive control (Figure 4d, lane 1). A clear DNA amplification was observed after immunoprecipitation with VDR antibody (Figure 4d, lane 3) but not with irrelevant IgG antibody (Figure 4d, lane 2). These findings provide a molecular mechanism underlying VDR‐dependent Nrf2 transcriptional activation.

The article "1,25‐Dihydroxyvitamin D exerts an antiaging role by activation of Nrf2‐antioxidant signaling and inactivation of p16/p53‐senescence signaling" was retracted in 2024. Reasons: manipulated images; errors in the images; duplicated images; unreliable data.

To determine whether the expression of antioxidant enzyme genes in the MEFs was dependent on Nrf2 or VDR, MEFs from wild‐type or VDR KO mice were transfected with small (short) interfering RNA (siRNA) which were Nrf2‐specific (siNrf2) and treated with or without 1,25(OH)_2_D_3_. Expression of Nrf2 mRNA was significantly reduced in MEFs transfected with Nrf2‐specific siRNA compared with MEFs transfected with control siRNA (Figure 4e). Furthermore, the expression levels of Nrf2 target genes, including GCS, GSR, Tmox1, and Cat, were decreased significantly in both wild‐type and VDR KO MEFs by Nrf2 silencing compared to the siRNA control. The target genes could be upregulated by 1,25(OH)_2_D_3_ treatment in wild‐type MEFs, but not in VDR KO MEFs (Figure 4f–i). Furthermore, in each case, this stimulation by 1,25(OH)_2_D_3_ was reduced by Nrf2 silencing demonstrating that a major portion of the effect of 1,25(OH)_2_D_3_ was via the action of Nrf2 (Figure 4f–i).

### 2.5 P16 deletion partly postpones aging induced by 1,25(OH)_2_D_3_deficiency

To assess whether p16 deletion can reduce aging arising from 1,25(OH)_2_D_3_deficiency, we examined compound mutant mice with homozygous deletion of both p16 and 1α(OH)ase [1α(OH)ase^−/−^p16^−/−^], and compared them to p16^−/−^, 1α(OH)ase^−/−^and their wild‐type littermates. The average lifespan of 1α(OH)ase^−/−^p16^−/−^ mice was significantly increased to 189 days (122–260 days) from the average 91 days that 1α(OH)ase^−/−^ mice survived (Figure 5a). Serum 1,25(OH)_2_D_3_and calcium and phosphorus levels were not different in wild‐type and p16^−/−^ mice, whereas serum 1,25(OH)_2_D_3_ was undetectable and serum calcium and phosphorus levels were decreased in both 1α(OH)ase^−/−^ and 1α(OH)ase^−/−^p16^−/−^ mice (Supporting Information Figure S5a–c). Body weight of 1α(OH)ase^−/−^p16^−/−^ mice was markedly elevated compared to 1α(OH)ase^−/−^ counterparts (Figure 5b). ROS levels in the skin and liver were increased dramatically in 1α(OH)ase^−/−^ mice; however, they were normalized in 1α(OH)ase^−/−^p16^−/−^ mice(Figure 5c and Supporting Information Figure S5d).The thickness of skin and collagen deposition in skin were not altered in p16^−/−^ mice and were decreased in 1α(OH)ase^−/−^ mice; however, they was increased significantly in 1α(OH)ase^−/−^p16^−/−^ mice compared with 1α(OH)ase^−/−^ mice (Figure 5d–g). The percentage of Ki67‐positive cells in the skin was decreased in both 1α(OH)ase^−/−^ and 1α(OH)ase^−/−^p16^−/−^ mice; however, the percentage was increased significantly in 1α(OH)ase^−/−^p16^−/−^ mice compared with 1α(OH)ase^−/−^ mice (Figure 5h,i). SA‐β‐gal‐positive areas in the skin, kidney, and lung (Figure 5j,k and Supporting Information Figure S5e–h) and SASP molecules including TNFα, IL‐1α and β, IL‐6, Mmp 3 and 13 in the skin, kidney, liver, and lung (Supporting Information Figure S5i–l) were not altered in p16^−/−^ mice and were increased dramatically in 1α(OH)ase^−/−^ mice compared with wild‐type mice; however, they were decreased significantly in 1α(OH)ase^−/−^p16^−/−^ mice compared with 1α(OH)ase^−/−^ mice. In addition, the protein expression levels of p53 and p21 in skin tissue were downregulated in p16^−/−^ mice and upregulated in 1α(OH)ase^−/−^ mice, whereas they were clearly downregulated in 1α(OH)ase^−/−^p16^−/−^ mice compared with 1α(OH)ase^−/−^ mice. In contrast, the protein expression levels of cyclinD1, cyclin E, and SOD2 were upregulated in p16^−/−^ mice and downregulated in 1α(OH)ase^−/−^mice, but were upregulated significantly in 1α(OH)ase^−/−^p16^−/−^ mice compared with 1α(OH)ase^−/−^ mice (Figure 5l,m). These findings demonstrated that p16 deletion can partly prevent aging resulting from 1,25(OH)_2_D_3_ deficiency by enhancing cell proliferative ability and reducing cell senescence and SASP.

The article "1,25‐Dihydroxyvitamin D exerts an antiaging role by activation of Nrf2‐antioxidant signaling and inactivation of p16/p53‐senescence signaling" was retracted in 2024. Reasons: manipulated images; errors in the images; duplicated images; unreliable data.

**Figure 5:** p16 deletion delays aging induced by 1,25(OH)_2_D_3_deficiency. (a) The survival rate of WT, p16^−/−^, 1α(OH)ase^−/−^, and 1α(OH)ase^−/−^p16^−/−^ mice; (b) body weight; (c) ROS levels in freshly isolated cells of skin; representative micrographs of skin sections from 10‐week‐old mice stained with (d) HE, (f) histochemically for total collagen and (h) immunohistochemically for Ki67 and (j) histochemically for SA‐β‐gal. Scale bars represent 200 μm in (d) and (f) and 50 μm in (h) and (j). (e) Skin thickness; (g) total collagen‐positive area; the percentage of (i) BrdU‐positive cells of skin; (k) the percentage of SA‐β‐gal‐positive area in skin; (l) representative Western blots of skin extracts to determine p53, p21, cyclin E, cyclin D1, and SOD protein levels in skin. β‐actin was used as loading control. (m) Skin protein levels relative to β‐actin protein levels were assessed by densitometric analysis and expressed as percentage of the levels of wild‐type mice. Each value is the means ± *SEM* of determinations in five mice of each group. *p < 0.05; ^**^ *p* < 0.01; ***p < 0.001 compared with WT mice. ^#^p* < *0.05; ^##^ *p < *0.01; ^###^ *p < *0.001 compared with 1α(OH)ase^−/−^ mice

The article "1,25‐Dihydroxyvitamin D exerts an antiaging role by activation of Nrf2‐antioxidant signaling and inactivation of p16/p53‐senescence signaling" was retracted in 2024. Reasons: manipulated images; errors in the images; duplicated images; unreliable data.

### 2.6 P53 haploinsufficiency partly postpones aging induced by 1,25(OH)_2_D_3_ deficiency

To explore whether p53 haploinsufficiency can postpone aging induced by 1,25(OH)_2_D_3_deficiency, we generated compound mutant mice that were homozygous for 1α(OH)ase deletion and heterozygous for p53 mutation (1α(OH)ase^−/−^p53^+/−^) and compared them to p53^+/−^, 1α(OH)ase^−/−^ and their wild‐type littermates. We found that the average lifespan was prolonged to 186 days (152–221 days) in 1α(OH)ase^−/−^p53^+/−^ mice from 90 days (66–120 days) in 1α(OH)ase^−/−^ mice, whereas the lifespan of the p53^+/−^ mice was longer than 10 months (Figure 6a). Serum 1,25(OH)_2_D_3_and calcium and phosphorus levels were not different from wild‐type in p53^+/−^ mice, whereas serum 1,25(OH)_2_D_3_ was undetectable and serum calcium and phosphorus levels were decreased in both 1α(OH)ase^−/−^ and 1α(OH)ase^−/−^p53^+/−^ mice (Supporting Information Figure S6a–c). Body size (Supporting Information Figure S6e) and body weight (Figure 6b) were increased in p53^+/−^mice and were decreased in both 1α(OH)ase^−/−^ and 1α(OH)ase^−/−^p53^+/−^ mice; however, they were increased significantly in 1α(OH)ase^−/−^p53^+/−^ mice compared with 1α(OH)ase^−/−^ mice. The thickness of skin and collagen deposition in skin were not altered in p53^+/−^ mice but were decreased in both 1α(OH)ase^−/−^ and 1α(OH)ase^−/−^p53^+/−^ mice; however, they were increased significantly in 1α(OH)ase^−/−^p53^+/−^ mice compared with 1α(OH)ase^−/−^ mice (Figure 6d–g). ROS levels in the skin (Figure 6c) and liver (Supporting Information Figure S6d) and γ‐H2AX‐positive cells in the skin (Figure 6h,i) were reduced in p53^+/−^ mice and were increased dramatically in 1α(OH)ase^−/−^ mice; however, they were normalized in 1α(OH)ase^−/−^p53^+/−^ mice. The percentage of Ki67‐positive cells in the skin was increased in p53^+/−^ mice and was decreased in both 1α(OH)ase^−/−^ and 1α(OH)ase^−/−^p53^+/−^ mice; however, it was increased significantly in 1α(OH)ase^−/−^p53^+/−^ mice compared with 1α(OH)ase^−/−^ mice (Figure 6j,k). SA‐β‐gal‐positive areas in the skin, kidney, and lung were not altered in p53^+/−^ mice and were increased dramatically 1α(OH)ase^−/−^ mice compared with wild‐type mice; however, they were decreased significantly in 1α(OH)ase^−/−^p53^+/−^ mice compared with1α(OH)ase^−/−^ mice (Figure 6l,m and Supporting Information Figure S6f–h). The percentage of TUNEL‐positive cells in skin were reduced in p53^+/−^ mice and increased dramatically 1α(OH)ase^−/−^ mice compared with wild‐type mice; however, they were decreased significantly in 1α(OH)ase^−/−^p53^+/−^ mice compared with in 1α(OH)ase^−/−^ mice (Figure 6o,p). Wnt 16, p53, p21, and caspase‐3 protein expression levels in the skin were all downregulated significantly in p53^+/−^ mice and upregulated dramatically in 1α(OH)ase^−/−^ mice; however, they were downregulated significantly in 1α(OH)ase^−/−^p53^+/−^ mice compared with in 1α(OH)ase^−/−^ mice (Figure 6q,r). In contrast, cyclin D1 and E were upregulated significantly in p53^+/−^ mice and downregulated dramatically in 1α(OH)ase^−/−^ mice, but were upregulated significantly in 1α(OH)ase^−/−^p53^+/−^ mice compared with1α(OH)ase^−/−^ mice (Figure 6q,r).These results demonstrated that p53 haploinsufficiency can partly postpone aging induced by 1,25(OH)_2_D_3_deficiency by inhibiting oxidative stress, DNA damage, cell senescence and apoptosis, and by stimulating cell proliferation.

The article "1,25‐Dihydroxyvitamin D exerts an antiaging role by activation of Nrf2‐antioxidant signaling and inactivation of p16/p53‐senescence signaling" was retracted in 2024. Reasons: manipulated images; errors in the images; duplicated images; unreliable data.

**Figure 6:** p53 haploinsufficiency delays aging induced by 1,25(OH)_2_D_3_deficiency. (a) The survival rates of WT, p53^+/−^, 1α(OH)ase^−/−^, and 1α(OH)ase^−/−^p53^+/−^ mice; (b) body weight; (c) ROS levels in freshly isolated cells of skin; representative micrographs of skin sections from 10‐week‐old mice stained with (d) HE, histochemically for (f) total collagen, immunohistochemically for (h) γ‐H2AX and (j) Ki‐67, histochemically for (l) SA‐β‐gal and (o) with TUNEL. Scale bars represent 200 μm in (d) and (f) and 50 μm in h, j, l, and o. (e) Skin thickness; (g) total collagen‐positive area; the percentage of (i) γ‐H2AX‐ and (k) Ki‐67‐positive cells of skin; (m) the percentage of SA‐β‐gal‐positive area in skin; (p) the percentage of TUNEL‐positive cells in skin. (q) Representative Western blots of skin extracts to determine Wnt16, p53, p21, caspase3, cyclin D1, and cyclin E protein levels in skin. β‐actin was used as loading control. (r) Skin protein levels relative to β‐actin protein levels were assessed by densitometric analysis and expressed as percentage of the levels of vehicle‐treated wild‐type mice fed the normal diet (ND). Each value is the mean ± *SEM* of determinations in five mice of each group. *p < 0.05; **p < 0.01; ***p < 0.001 compared with WT mice. *^#^p < *0.05; *^##^p <* 0.01; ^###^ *p* *<* 0.001 compared with 1α(OH)ase^−/−^ mice

## 3 DISCUSSION

In the present study, we first compared the effects on lifespan, of 1,25(OH)_2_D_3_deficiency alone, or after supplementation with high calcium/phosphate, supplementation with combined calcium/phosphate and antioxidant NAC, or supplementation with exogenous 1,25(OH)_2_D_3_. We found that the average lifespan of 1,25(OH)_2_D_3‐_deficient mice was only 91 days when fed a normal diet, was prolonged to 252 days when fed a high calcium/phosphate diet, and was further prolonged to 487 days when they were supplemented with exogenous 1,25(OH)_2_D_3._The average lifespan was 409 days when they were supplemented with combined calcium/phosphate and antioxidant NAC, which was clearly greater than with the high calcium/phosphate diet alone, but was not as long as when supplemented with exogenous 1,25(OH)_2_D_3_. These results indicate that 1,25(OH)_2_D_3_deficiency could reduce lifespan, whereas exogenous 1,25(OH)_2_D_3_supplementation could prolong the lifespan mediated via its function to maintain both calcium/phosphate and redox balance. Excess exogenous 1,25(OH)_2_D_3_ supplementation could however lead to hypercalcemia.

The article "1,25‐Dihydroxyvitamin D exerts an antiaging role by activation of Nrf2‐antioxidant signaling and inactivation of p16/p53‐senescence signaling" was retracted in 2024. Reasons: manipulated images; errors in the images; duplicated images; unreliable data.

We found that normalization of serum calcium/phosphate levels by supplementation with calcium/phosphate not only prolonged the lifespan of 1,25(OH)_2_D_3‐_deficient mice, but also improved their growth and aging phenotypes. Thus, supplementation with calcium/phosphate significantly reduced oxidative stress, DNA damage, senescence cells, and SASP molecule levels in multiple organs of 1,25(OH)_2_D_3‐_deficient mice. Moreover, combined supplementation of calcium/phosphate and antioxidant NAC not only further extended the lifespan of 1,25(OH)_2_D_3‐_deficient mice, but also more markedly improved organismal aging phenotypes induced by 1,25(OH)_2_D_3_deficiency, that is, they reduced oxidative stress, DNA damage, senescence cells, and SASP molecule levels, and also augmented cell proliferation by upregulating expression levels of the oncogene Bmi1 and downregulating expression of p16, p53, and p21. When comparing the effects of supplementation of combined calcium/phosphate and antioxidant NAC in preventing aging, with those of supplementation of exogenous 1,25(OH)_2_D_3,_we found that their roles were almost comparable in inhibiting oxidative stress, DNA damage, cell senescence and SASP, and stimulating cell proliferation with upregulation of Bmi1 and downregulation of p16, p53, and p21. However, supplementation of exogenous 1,25(OH)_2_D_3_mice more significantly extended the lifespan of 1,25(OH)_2_D_3‐_deficient mice than did supplementation with combined calcium/phosphate and antioxidant NAC. Our results imply that 1,25(OH)_2_D_3_can postpone aging mainly by maintaining both calcium/phosphate and redox balances_._

The role and mechanism of 1,25(OH)_2_D in maintaining calcium and phosphorus balance has been extensively studied (Fleet, 2017; Veldurthy et al., 2016). However, the mechanism of action of 1,25(OH)_2_D in maintaining the redox balance is not yet clear. Previous studies have shown that 1,25(OH)_2_D_3_reduced oxidative stress in human prostate epithelial cells (Bao, Ting, Hsu, & Lee, 2008) and human endothelial cells by activation of Nrf2‐antioxidant Signals (Moi et al., 1994). However, it is unclear whether 1,25(OH)_2_D_3_exerts an antioxidant role by transcriptional regulation of Nrf2 mediated through VDR. In this study, we demonstrated that Nrf2 expression levels were upregulated significantly in 1,25(OH)_2_D_3_‐treated MEFs from wild‐type mice in a dose‐dependent manner, but not in these from VDR knockout mice. The putative promoter region containing the predicted VDR binding sites of the Nrf2 gene was suggested by bioinformatic analysis and luciferase assays demonstrated that the putative promoter region containing the predicted VDR binding sites of the Nrf2 gene is sufficient to promote transcription of Nrf2, and Nrf2 transcription was further enhanced by 1,25(OH)_2_D_3_treatment. Furthermore, we showed that the VDR has the ability to physically bind the Nrf2 promoter using a ChIP approach. We also demonstrated that Nrf2 knockdown reduced the expression levels of Nrf2 target genes including Nqo1, GCS, Cat, Txnrd1, and Sod1. Taken together, our results indicate that 1,25(OH)_2_D_3_exerts an antioxidant role in large part by transcriptional regulation of Nrf2 mediated through the VDR.

The article "1,25‐Dihydroxyvitamin D exerts an antiaging role by activation of Nrf2‐antioxidant signaling and inactivation of p16/p53‐senescence signaling" was retracted in 2024. Reasons: manipulated images; errors in the images; duplicated images; unreliable data.

Induction of cellular senescence occurs at least in part through redox‐dependent activation of the p38‐p16 pathway (Ito et al., 2006). Chronic oxidative stress activates p38 signaling and blocks Akt‐dependent stabilization of Bmi1 (a negative regulator of the Ink4a/Arf locus), resulting in accelerated proteasome‐mediated degradation of Bmi1 (Kim, Hwangbo, & Wong, 2011), whereas Bmi1 loss has been shown to induce mitochondrial dysfunction directly and also induce upregulation of p16/ARF (Liu et al., 2009). Our results demonstrated that 1,25(OH)_2_D_3_deficiency not only increased ROS levels and DNA damage and upregulated p53 and p21 expression levels, but also upregulated p16 and downregulated Bmi1 expression levels. We also found that tissue cell senescence and SASP inhibited by supplementation with exogenous 1,25(OH)_2_D_3_or with combined calcium/phosphate and antioxidant NAC was associated with downregulation of p16 and upregulation of Bmi1. These results suggest that p16 is another critical downstream target of 1,25(OH)_2_D_3._To further demonstrate this, we deleted p16 in 1α(OH)ase^−/−^ mice and found that p16 deletion not only significantly prolonged their lifespan, but also rescued their aging phenotypes by enhancing cell proliferative ability and reducing cell senescence and SASP. Previous studies showed that removing p16^Ink4a^‐expressing senescent cells from a mouse model of accelerated aging delays the onset of several aging disease‐related processes (Baker et al., 2011). Recently, it has also been reported that the elimination of p16^Ink4a^‐expressing cells from of wild‐type mice increased lifespan and ameliorated a range of age‐dependent, disease‐related abnormalities, suggesting that the accumulation of p16^Ink4a^‐expressing cells during aging shortens lifespan (Baker et al., 2016). Our results demonstrated that ablation of p16 could extend the lifespan of 1,25(OH)_2_D_3_ deficient mice. Although it has been reported that p16 may not directly be involved in the induction of SASP, and that activation of the DNA damage‐induced stimulator of interferon genes (STING) pathway induces SASP (Takahashi et al., 2018), recent studies have also shown that induction of p16, for example, by loss of H3K27me3 is associated with activation of SASP although this did appear to be independent of DNA damage (Ito, Teo, Evans, Neretti, & Sedivy, 2018). Therefore, it is possible that a decrease in 1,25(OH)_2_D_3_ induced an increase in p16 as well as DNA damage both of which independently contribute to increased SASP.

The article "1,25‐Dihydroxyvitamin D exerts an antiaging role by activation of Nrf2‐antioxidant signaling and inactivation of p16/p53‐senescence signaling" was retracted in 2024. Reasons: manipulated images; errors in the images; duplicated images; unreliable data.

We also found that 1,25(OH)_2_D_3_deficiency not only increased oxidative stress, but also increased DNA damage and activated p53‐p21 signaling, whereas supplementation with exogenous 1,25(OH)_2_D_3_or combined calcium/phosphate and antioxidant NAC administration not only inhibited oxidative stress, but also reduced DNA damage and downregulated p53 and p21 expression levels. Therefore, we asked whether p53 knockdown could rescue aging phenotypes induced by 1,25(OH)_2_D_3_deficiency. In view of the fact that homozygous p53 mutants die at an early age from cancer (Donehower et al., 1992), we generated compound mutant mice that were homozygous for 1α(OH)ase deletion and heterozygous for p53 mutation and compared their phenotypes with 1,25(OH)_2_D_3‐_deficient mice. Our results demonstrated that p53 haploinsufficiency can partly postpone aging induced by 1,25(OH)_2_D_3_deficiency by inhibiting oxidative stress, DNA damage, cell senescence and apoptosis and by stimulating cell proliferation. Early evidence linking p53 to aging arose from the analysis of a mutant mouse model with an aberrant truncation of the N‐terminal portion of the protein. The truncated mutant proteins showed a robust constitutive p53 activity, and the mutant mice presented an array of aging‐related features and severely reduced lifespan (Tyner et al., 2002). Scrable and colleagues described a transgenic mouse overexpressing a modestly truncated, naturally occurring isoform of p53 called p44 that exhibited reduced lifespan, early bone loss, reduced body mass, premature loss of fertility and testicular degeneration, and altered IGF‐1 signaling (Maier et al., 2004). These results led to the notion that excessive p53 activity compromises healthy aging (Rufini et al., 2013). On the other hand, whether lack of reduced intact p53 activity affects lifespan has been difficult to assess, because of the severe tumor phenotype that accompanies loss of intact p53 (Donehower et al., 1992). Our study demonstrated that 1,25(OH)_2_D_3_deficiency accelerated aging with excessive p53 expression, whereas reducing p53 expression levels in 1,25(OH)_2_D_3‐_deficient mice by heterozygous deletion of p53 can clearly prolong lifespan. Our results support the observations that p53 functions are involved in cell‐cycle control, DNA repair, apoptosis, and cellular stress responses. In addition to inducing cell growth arrest and apoptosis, p53 activation also modulates cellular senescence and organismal aging. Our results therefore suggest that p53 is an important downstream target of 1,25(OH)_2_D_3_for preventing aging.

The article "1,25‐Dihydroxyvitamin D exerts an antiaging role by activation of Nrf2‐antioxidant signaling and inactivation of p16/p53‐senescence signaling" was retracted in 2024. Reasons: manipulated images; errors in the images; duplicated images; unreliable data.

Overall, therefore, the results of this study provide a model that suggests that 1,25(OH)_2_D_3_deficiency results in increasing oxidative stress through inhibiting transcription of Nrf2 and enhancing DNA damage; in addition, activation of p16/Rb and p53/p21 signaling occurs. These events then lead to inhibition of cellular proliferation and induction of cellular senescence and SASP, and thus acceleration of aging (Figure 7). These processes may be rescued to different degrees and aging postponed by supplementation of exogenous 1,25(OH)_2_D_3_, calcium/phosphate alone or combined calcium/phosphate and antioxidant NAC, or knockdown of p53 or knockout of p16 (Figure 7). This study not only identifies novel mechanisms of 1,25(OH)_2_D_3_deficiency in accelerating aging, but may also provide experimental and theoretical evidence for potential utilization of 1,25(OH)_2_D_3_or downstream targets to delay aging.

**Figure 7:** Model of mechanisms leading from 1,25(OH)_2_D_3_ deficiency to accelerated aging

## 4 EXPERIMENTAL PROCEDURES

### 4.1 Animals and treatments

The generation and characterization of 1α(OH)ase^−/−^ mice were previously described by us (Panda et al., 2001) and were generated on a BALB/c background. 1α(OH)ase^−/−^ mice were generated through breeding of heterozygous (1α(OH)ase^+/−^) mice and identified by PCR with tail genomic DNA as the template. Wild‐type littermates were used as controls in all the experiments.

One hundred and twenty pairs of age‐ and gender‐matched 1α(OH)ase^−/−^ and wild‐type littermates were randomly divided into four groups. After weaning, sex‐matched wild‐type and 1α(OH)ase^−/−^ mice were weaned onto one of the following four different regimens: (a) a normal diet (ND): containing 1.0% calcium, 0.67% phosphorus, and 2.2 IU vitamin D/g; (b) a rescue diet (RD, TD96348 Teklad, Madison, WI): containing 2.0% calcium, 1.25% phosphorus, 20% lactose, and 2.2 IU vitamin D/g; (c) a 1,25(OH)_2_D_3_supplemented diet (VD), that is, a normal diet plus thrice weekly subcutaneous injections of 1,25(OH)_2_D_3_ at a dose of 1 μg/kg per mouse; and (d) a NAC‐supplemented diet (RD + NAC), that is, a rescue diet plus 1 mg/ml *N*‐acetylcysteine (NAC) in drinking water. Five pairs of 10‐week‐old gender‐matched 1α(OH)ase^−/−^ and wild‐type littermates per group were used for phenotype analysis, and 25 pairs per group were maintained until death or until 600 days of age and were used for monitoring lifespan.

1α(OH)ase^+/−^mice, originally on a BALB/c background, were repeatedly backcrossed with wild‐type mice on a C57BL/6J background for 12 generations to obtain 1α(OH)ase^+/−^ mice on a C57BL/6J background. The 1α(OH)ase^+/−^ mice and p53^+/−^ mice (on a C57BL/6J background, purchased from Jackson Laboratory) or p16^+/−^mice (on a C57BL/6J background, purchased from Jackson Laboratory) were fertile and were mated to produce offspring heterozygous at both loci, which were then mated to generate 1α(OH)ase^−/−^p53^+/−^ or 1α(OH)ase^−/−^p16^−/−^pups. In the current study, 10‐week‐old wild‐type, p53^+/−^, 1α(OH)ase^−/−^, and 1α(OH)ase^−/−^p53^+/−^ mice or wild‐type, p16^−/−^, 1α(OH)ase^−/−^, and 1α(OH)ase^−/−^p16^−/−^ mice were used for phenotype analysis and others were maintained until 1 year of age for monitoring lifespan.

The article "1,25‐Dihydroxyvitamin D exerts an antiaging role by activation of Nrf2‐antioxidant signaling and inactivation of p16/p53‐senescence signaling" was retracted in 2024. Reasons: manipulated images; errors in the images; duplicated images; unreliable data.

All animal experiments were carried out in compliance with, and approval by, the Institutional Animal Care and Use Committee of Nanjing Medical University.

### 4.2 Measurements of serum calcium, phosphorus, and 1,25(OH)_2_D_3_

Serum calcium and phosphorus levels were analyzed by an autoanalyzer (Beckman Synchron 67; Beckman Instruments). Serum 1,25(OH)_2_D_3_ and 25(OH)D levels were measured by radioimmunoassay (Diagnostic Products, Los Angeles, CA), whereas serum intact PTH was measured with an ELISA (Immutopics, Inc., San Clemente, CA).

### 4.3 RNA isolation and real‐time RT–PCR

RNA was isolated from mouse skin, lung, liver, kidney, and spleen using TRIzol reagent (Invitrogen, Carlsbad, CA, USA) according to the manufacturer's protocol. Real‐time RT–PCR was performed as described previously (Zhou et al., 2016), and the primer sequences used for the real‐time PCR are presented in Supporting Information Table S1.

### 4.4 Histology

Skin, liver, kidney, and lung were removed and fixed in PLP fixative overnight at 4°C and processed histologically as we previously described (Miao et al., 2008). Afterward, tissues were dehydrated and embedded in paraffin, following which 5‐µm sections were cut on a rotary microtome. The sections were stained histochemically for total collagen and senescence‐associated‐β‐galactosidase (SA‐β‐gal) as previously described (Dimri et al., 1995), and immunohistochemically as described below.

The article "1,25‐Dihydroxyvitamin D exerts an antiaging role by activation of Nrf2‐antioxidant signaling and inactivation of p16/p53‐senescence signaling" was retracted in 2024. Reasons: manipulated images; errors in the images; duplicated images; unreliable data.

### 4.5 Immunohistochemistry

Immunohistochemical staining was carried out for Ki‐67, phosphorylation of histone H2AX on Ser139 (γ‐H2AX), and superoxide dismutase 2 (SOD2) using the avidin–biotin–peroxidase complex technique with affinity‐purified rabbit polyclonal antibody against Ki‐67 (ab16667; Abcam), rabbit polyclonal antibody against γ‐H2AX (#9718; Cell Signaling Technology), and rabbit polyclonal antibody against SOD2 (NB100‐1992; Novus Biological). Briefly, dewaxed and rehydrated paraffin‐embedded sections were incubated with methanol: hydrogen peroxide (1:10) to block endogenous peroxidase activity and then washed in Tris‐buffered saline (pH 7.6). Slides were then incubated with the primary antibodies overnight at room temperature. After rinsing with Tris‐buffered saline for 15 min, tissues were incubated with secondary antibody (biotinylated goat anti‐rabbit IgG; Sigma). Sections were then washed and incubated with the Vectastain Elite ABC reagent (Vector Laboratories) for 45 min. Staining was developed using 3,3‐diaminobenzidine (2.5 mg/ml) followed by counterstaining with Mayer's hematoxylin.

### 4.6 Computer‐assisted image analysis

Sections stained histochemically or immunohistochemically were photographed under a Leica DM4000B photomicroscope (Leica, Wetzlar, Germany) and analyzed with Northern Eclipse image analysis software (Empix Imaging Inc., Mississauga, ON, Canada) as described (Jiang et al., 2015). All image analyses were based on a high power field (40× obj.) except for measuring the skin thickness in H&E‐stained sections (20× obj.). Skin thickness including epidermal and dermal skin with subcutaneous tissue was measured. The positive areas for histochemical or immunohistochemical positive products were expressed as the percentages of total skin areas. The immunopositive cell numbers were averaged and expressed as the percentage of positive cells of total cell numbers.

### 4.7 Western blot

Proteins were extracted from the skin or liver of each group of mice. Immunoblotting was carried out as previously described (Miao et al., 2008). Primary antibodies against peroxiredoxin‐I (PrdxI) (sc‐7381; Santa Cruz Biotechnology), Bmi1 (05‐637; Millipore), p16 (sc‐377412; Santa Cruz Biotechnology), p53 (#2524; Cell Signaling Technology), p21 (sc‐471; Santa Cruz Biotechnology), Wnt16 (sc‐20964, Santa Cruz Biotechnology), caspase‐3 (#9662; Cell signaling technology), cyclin D1 (#2922; Cell signaling technology), cyclin E (sc‐377100; Santa Cruz Biotechnology), and β‐actin (AP0060; Bioworld Technology) were used. Immunoreactive bands were visualized with ECL chemiluminescence (Amersham) and analyzed by Scion Image Beta 4.02 (Scion, National Institutes of Health).

The article "1,25‐Dihydroxyvitamin D exerts an antiaging role by activation of Nrf2‐antioxidant signaling and inactivation of p16/p53‐senescence signaling" was retracted in 2024. Reasons: manipulated images; errors in the images; duplicated images; unreliable data.

### 4.8 Intracellular ROS analysis

For analysis of intracellular ROS, tissues from skin, liver, or kidney were trypsinized, converted into single cell suspensions, washed with cold PBS, and resuspended in a binding buffer. 10^6^ cells of skin, liver, or kidney from 10‐week‐old mice were incubated with 5 mM diacetyldichlorofluorescein (DCFDA; Invitrogen) and placed in a shaker at 37°C for 30 min, followed immediately by flow cytometry analysis in a FACS Calibur flow cytometer (Becton Dickinson, Heidelberg, Germany).

### 4.9 TUNEL assay

Dewaxed and rehydrated paraffin sections were stained with an In Situ Cell Death Detection kit (Roche Diagnostics Corp., Basel, Switzerland) using a previously described protocol (Jin et al., 2011).

### 4.10 Isolation and cultures of mouse embryonic fibroblasts

Wild‐type and VDR^−/−^ female mice (on a C57BL/6J background, a generous gift of Dr. Marie Demay, Massachusetts General Hospital, Boston, MA) at day 13.5 of gestation were used for isolation of mouse embryonic fibroblasts (MEFs). All mice were anesthetized with 2% chloral hydrate and killed by cervical dislocation; embryos were removed from the uterus and were collected in the transfer media containing DMEM and 1% penicillin/streptomycin antibiotics, and then fetal liver, head, and residual limbs were removed. The embryos were washed with PBS. The tissues were triturated in 0.05% Trypsin‐EDTA (1X) and digested for 20 min, mixing well every 5 min. The enzyme activity was naturalized with FBS, and cell suspensions were transferred to DMEM containing 10% FBS and cultured in an incubator at 37°C in a 5% CO_2_ atmosphere.

### 4.11 Plasmid constructs and luciferase reporter assay

Using mouse genomic DNA as a template, PCR was used to amplify the whole Nrf2 promoter segment −613 to −361. The PCR products with the predicted wild‐type VDR binding site “aggttctgcaggtcca and with a mutated site (Figure 4b), synthesized by Shandong Weizhen Biotechnology Co., Ltd., were then cloned into pGL3‐basic vectors to obtain Nrf2‐PGL3 and Nrf2‐PGL3 mutant plasmids. MEF cells were transfected with VDR‐Pcdn3.1 and Nrf2‐PGL3 or mutant‐Nrf2‐PGL3 plasmids in 24‐well plates using Lipofectamine 2000 (Invitrogen) according to the manufacturer's instructions and then incubated with normal medium, with or without 10^−7^ M 1,25(OH)_2_D_3_ (D1530‐; Sigma). Forty‐eight hours after transfection, the cells were harvested and lysed for luciferase assays. The relative luciferase activity was normalized to Renilla luciferase activity.

The article "1,25‐Dihydroxyvitamin D exerts an antiaging role by activation of Nrf2‐antioxidant signaling and inactivation of p16/p53‐senescence signaling" was retracted in 2024. Reasons: manipulated images; errors in the images; duplicated images; unreliable data.

### 4.12 Chromatin immunoprecipitation assays

Chromatin immunoprecipitation (ChIP) assays were performed using the CHIP kit according to the manufacturer's instructions (Cell signaling technology, #9004, USA). VDR antibody was obtained from Abcam (ab3508). The ChIP primer sequence was designed by Primer Premier 5: Nrf2 sense 5′‐TGGGGCAGAGGTGTTTGAGC‐3′ and antisense 5′‐CCCTGGCTCTTTGAAGCAGTTTA‐3′. The relative binding of VDR to Nrf2 was determined through PCR by digital imaging system gel exposure on agarose gels.

### 4.13 Nrf2 knockdown

The Nrf2 siRNA was a gift from Professor Shizhong Zheng (Nanjing University of Chinese Medicine). SiNrf2 (100 nM) and control siRNA (100 nM) were transfected into MEFs using Lipofectamine 2000 (Invitrogen) according to the manufacturer's instructions. The transfected medium was removed after 4–6 hr and then replaced with the normal medium in the absence or presence of 10^−7^ M 1,25(OH)_2_D_3_. Cells were collected for real‐time RT–PCR analyses 48 hr after transfections.

### 4.14 Statistical analysis

All analyses were performed using SPSS software (Version 16.0, SPSS Inc., Chicago, IL, USA). Measured data were described as mean ± *SEM* and analyzed by Student's *t* test and one‐way ANOVA to compare differences between groups. Qualitative data were described as percentages and analyzed using a chi‐square test as indicated. *p* values were two‐sided, and <0.05 was considered statistically significant.

## CONFLICT OF INTEREST

None declared.

## AUTHOR CONTRIBUTIONS

D.M. and D.G. conceived the project. L.C., R.Y., W.Q., and W.Z. performed most of the experiments, analyzed, and compiled the data. J.C. and L.M. helped with experiments. D.M., D.G., L.C., and R.Y. participated in writing or editing the paper.

## References

[acel12951-bib-0001] Baker, D. J. , Childs, B. G. , Durik, M. , Wijers, M. E. , Sieben, C. J. , Zhong, J. , … van Deursen, J. M. (2016). Naturally occurring p16(Ink4a)‐positive cells shorten healthy lifespan. Nature, 530, 184–189. 10.1038/nature16932 26840489PMC4845101

[acel12951-bib-0002] Baker, D. J. , Wijshake, T. , Tchkonia, T. , LeBrasseur, N. K. , Childs, B. G. , van de Sluis, B. , … van Deursen, J. M. (2011). Clearance of p16Ink4a‐positive senescent cells delays ageing‐associated disorders. Nature, 479, 232–236. 10.1038/nature10600 22048312PMC3468323

[acel12951-bib-0003] Bao, B. Y. , Ting, H. J. , Hsu, J. W. , & Lee, Y. F. (2008). Protective role of 1 alpha, 25‐dihydroxyvitamin D3 against oxidative stress in nonmalignant human prostate epithelial cells. International Journal of Cancer, 122, 2699–2706.1834814310.1002/ijc.23460

[acel12951-bib-0004] Berridge, M. J. (2015a). Vitamin D cell signalling in health and disease. Biochemical and Biophysical Research Communications, 460, 53–71.2599873410.1016/j.bbrc.2015.01.008

[acel12951-bib-0005] Berridge, M. J. (2015b). Vitamin D: A custodian of cell signalling stability in health and disease. Biochemical Society Transactions, 43, 349–358.2600917510.1042/BST20140279

[acel12951-bib-0006] Cheung, K. L. , Lee, J. H. , Khor, T. O. , Wu, T. Y. , Li, G. X. , Chan, J. , … Kong, A. N. (2014). Nrf2 knockout enhances intestinal tumorigenesis in Apc(min/+) mice due to attenuation of anti‐oxidative stress pathway while potentiates inflammation. Molecular Carcinogenesis, 53, 77–84.2291189110.1002/mc.21950

[acel12951-bib-0007] Dimri, G. P. , Lee, X. , Basile, G. , Acosta, M. , Scott, G. , Roskelley, C. , … Pereira‐Smith, O. (1995). A biomarker that identifies senescent human cells in culture and in aging skin in vivo. Proceedings of the National Academy of Sciences of the United States of America, 92, 9363–9367. 10.1073/pnas.92.20.9363 7568133PMC40985

[acel12951-bib-0008] Donehower, L. A. , Harvey, M. , Slagle, B. L. , McArthur, M. J. , Montgomery, C. A., Jr. , Butel, J. S. , & Bradley, A. (1992). Mice deficient for p53 are developmentally normal but susceptible to spontaneous tumours. Nature, 356, 215–221. 10.1038/356215a0 1552940

[acel12951-bib-0009] Fleet, J. C. (2017). The role of vitamin D in the endocrinology controlling calcium homeostasis. Molecular and Cellular Endocrinology, 453, 36–45. 10.1016/j.mce.2017.04.008 28400273PMC5529228

[acel12951-bib-0010] Halicka, H. D. , Zhao, H. , Li, J. , Traganos, F. , Studzinski, G. P. , & Darzynkiewicz, Z. (2012). Attenuation of constitutive DNA damage signaling by 1,25‐dihydroxyvitamin D3. Aging, 4, 270–278. 10.18632/aging.100450 22498490PMC3371762

[acel12951-bib-0011] Haussler, M. R. , Haussler, C. A. , Whitfield, G. K. , Hsieh, J. C. , Thompson, P. D. , Barthel, T. K. , … Jurutka, P. W. (2010). The nuclear vitamin D receptor controls the expression of genes encoding factors which feed the "Fountain of Youth" to mediate healthful aging. Journal of Steroid Biochemistry and Molecular Biology, 121, 88–97. 10.1016/j.jsbmb.2010.03.019 20227497PMC2906618

[acel12951-bib-0012] Haussler, M. R. , Whitfield, G. K. , Haussler, C. A. , Sabir, M. S. , Khan, Z. , Sandoval, R. , & Jurutka, P. W. (2016). 1,25‐Dihydroxyvitamin D and Klotho: A tale of two renal hormones coming of age. Vitamins and Hormones, 100, 165–230.2682795310.1016/bs.vh.2015.11.005

[acel12951-bib-0013] Hayes, J. D. , & Dinkova‐Kostova, A. T. (2014). The Nrf2 regulatory network provides an interface between redox and intermediary metabolism. Trends in Biochemical Sciences, 39, 199–218. 10.1016/j.tibs.2014.02.002 24647116

[acel12951-bib-0014] Ito, K. , Hirao, A. , Arai, F. , Takubo, K. , Matsuoka, S. , Miyamoto, K. , … Suda, T. (2006). Reactive oxygen species act through p38 MAPK to limit the lifespan of hematopoietic stem cells. Nature Medicine, 12, 446–451. 10.1038/nm1388 16565722

[acel12951-bib-0015] Ito, T. , Teo, Y. V. , Evans, S. A. , Neretti, N. , & Sedivy, J. M. (2018). Regulation of cellular senescence by polycomb chromatin modifiers through distinct DNA damage‐ and histone methylation‐dependent pathways. Cell Reports, 22, 3480–3492. 10.1016/j.celrep.2018.03.002 29590617PMC5915310

[acel12951-bib-0016] Javanbakht, M. (2010). The effects of vitamins E and D supplementation on erythrocyte superoxide dismutase and catalase in atopic dermatitis. Iranian Journal of Public Health, 39, 57–63.23112990PMC3468963

[acel12951-bib-0017] Jiang, M. , Chen, G. , Lu, N. , Zhang, Y. , Jin, S. , Karaplis, A. , … Miao, D. (2015). Deficiency of the parathyroid hormone‐related peptide nuclear localization and carboxyl terminal sequences leads to premature skin ageing partially mediated by the upregulation of p27. Experimental Dermatology, 24, 847–852. 10.1111/exd.12789 26121068

[acel12951-bib-0018] Jin, J. , Zhao, Y. , Tan, X. , Guo, C. , Yang, Z. , & Miao, D. (2011). An improved transplantation strategy for mouse mesenchymal stem cells in an acute myocardial infarction model. PloS One, 6, e21005 10.1371/journal.pone.0021005 21698117PMC3117862

[acel12951-bib-0019] Keisala, T. , Minasyan, A. , Lou, Y. R. , Zou, J. , Kalueff, A. V. , Pyykko, I. , & Tuohimaa, P. (2009). Premature aging in vitamin D receptor mutant mice. Journal of Steroid Biochemistry and Molecular Biology, 115, 91–97. 10.1016/j.jsbmb.2009.03.007 19500727

[acel12951-bib-0020] Kim, J. , Hwangbo, J. , & Wong, P. K. (2011). p38 MAPK‐Mediated Bmi‐1 down‐regulation and defective proliferation in ATM‐deficient neural stem cells can be restored by Akt activation. PloS One, 6, e16615 10.1371/journal.pone.0016615 21305053PMC3030607

[acel12951-bib-0021] Krishnamurthy, J. , Torrice, C. , Ramsey, M. R. , Kovalev, G. I. , Al‐Regaiey, K. , Su, L. , & Sharpless, N. E. (2004). Ink4a/Arf expression is a biomarker of aging. Journal of Clinical Investigation, 114, 1299–1307. 10.1172/JCI22475 15520862PMC524230

[acel12951-bib-0022] Kubben, N. , Zhang, W. , Wang, L. , Voss, T. C. , Yang, J. , Qu, J. , … Misteli, T. (2016). Repression of the antioxidant NRF2 pathway in premature aging. Cell, 165, 1361–1374. 10.1016/j.cell.2016.05.017 27259148PMC4893198

[acel12951-bib-0023] Li, Y. C. , Pirro, A. E. , Amling, M. , Delling, G. , Baron, R. , Bronson, R. , & Demay, M. B. (1997). Targeted ablation of the vitamin D receptor: An animal model of vitamin D‐dependent rickets type II with alopecia. Proceedings of the National Academy of Sciences of the United States of America, 94, 9831–9835.927521110.1073/pnas.94.18.9831PMC23277

[acel12951-bib-0024] Lin, A. M. , Chen, K. B. , & Chao, P. L. (2005). Antioxidative effect of vitamin D3 on zinc‐induced oxidative stress in CNS. Annals of the New York Academy of Sciences, 1053, 319–329. 10.1196/annals.1344.028 16179538

[acel12951-bib-0025] Liu, J. , Cao, L. , Chen, J. , Song, S. , Lee, I. H. , Quijano, C. , … Finkel, T. (2009). Bmi1 regulates mitochondrial function and the DNA damage response pathway. Nature, 459, 387–392. 10.1038/nature08040 19404261PMC4721521

[acel12951-bib-0026] Maier, B. , Gluba, W. , Bernier, B. , Turner, T. , Mohammad, K. , Guise, T. , … Scrable, H. (2004). Modulation of mammalian life span by the short isoform of p53. Genes & Development, 18, 306–319. 10.1101/gad.1162404 14871929PMC338283

[acel12951-bib-0027] Miao, D. , Su, H. , He, B. , Gao, J. , Xia, Q. , Zhu, M. , … Karaplis, A. C. (2008). Severe growth retardation and early lethality in mice lacking the nuclear localization sequence and C‐terminus of PTH‐related protein. Proceedings of the National Academy of Sciences of the United States of America, 105, 20309–20314. 10.1073/pnas.0805690105 19091948PMC2629292

[acel12951-bib-0028] Moi, P. , Chan, K. , Asunis, I. , Cao, A. , & Kan, Y. W. (1994). Isolation of NF‐E2‐related factor 2 (Nrf2), a NF‐E2‐like basic leucine zipper transcriptional activator that binds to the tandem NF‐E2/AP1 repeat of the beta‐globin locus control region. Proceedings of the National Academy of Sciences of the United States of America, 91, 9926–9930. 10.1073/pnas.91.21.9926 7937919PMC44930

[acel12951-bib-0029] Mokry, L. E. , Ross, S. , Ahmad, O. S. , Forgetta, V. , Smith, G. D. , Goltzman, D. , … Richards, J. B. (2016). Correction: Vitamin D and risk of multiple sclerosis: A Mendelian randomization study. PLoS Med, 13, e1001981 10.1371/journal.pmed.1001981 26963823PMC4775038

[acel12951-bib-0030] Panda, D. K. , Miao, D. , Bolivar, I. , Li, J. , Huo, R. , Hendy, G. N. , & Goltzman, D. (2004). Inactivation of the 25‐hydroxyvitamin D 1alpha‐hydroxylase and vitamin D receptor demonstrates independent and interdependent effects of calcium and vitamin D on skeletal and mineral homeostasis. Journal of Biological Chemistry, 279, 16754–16766.1473929610.1074/jbc.M310271200

[acel12951-bib-0031] Panda, D. K. , Miao, D. , Tremblay, M. L. , Sirois, J. , Farookhi, R. , Hendy, G. N. , & Goltzman, D. (2001). Targeted ablation of the 25‐hydroxyvitamin D 1alpha ‐hydroxylase enzyme: Evidence for skeletal, reproductive, and immune dysfunction. Proceedings of the National Academy of Sciences of the United States of America, 98, 7498–7503.1141622010.1073/pnas.131029498PMC34697

[acel12951-bib-0032] Rai, P. , Onder, T. T. , Young, J. J. , McFaline, J. L. , Pang, B. , Dedon, P. C. , & Weinberg, R. A. (2009). Continuous elimination of oxidized nucleotides is necessary to prevent rapid onset of cellular senescence. Proceedings of the National Academy of Sciences of the United States of America, 106, 169–174. 10.1073/pnas.0809834106 19118192PMC2629241

[acel12951-bib-0033] Richards, J. B. , Valdes, A. M. , Gardner, J. P. , Paximadas, D. , Kimura, M. , Nessa, A. , … Aviv, A. (2007). Higher serum vitamin D concentrations are associated with longer leukocyte telomere length in women. American Journal of Clinical Nutrition, 86, 1420–1425. 10.1093/ajcn/86.5.1420 17991655PMC2196219

[acel12951-bib-0034] Rufini, A. , Tucci, P. , Celardo, I. , & Melino, G. (2013). Senescence and aging: The critical roles of p53. Oncogene, 32, 5129–5143. 10.1038/onc.2012.640 23416979

[acel12951-bib-0035] Smith, D. C. , Johnson, C. S. , Freeman, C. C. , Muindi, J. , Wilson, J. W. , & Trump, D. L. (1999). A Phase I trial of calcitriol (1,25‐dihydroxycholecalciferol) in patients with advanced malignancy. Clinical Cancer Research: an Official Journal of the American Association for Cancer Research, 5, 1339–1345.10389917

[acel12951-bib-0036] Takahashi, A. , Loo, T. M. , Okada, R. , Kamachi, F. , Watanabe, Y. , Wakita, M. , … Hara, E. (2018). Downregulation of cytoplasmic DNases is implicated in cytoplasmic DNA accumulation and SASP in senescent cells. Nature Communications, 9, 1249 10.1038/s41467-018-03555-8 PMC587185429593264

[acel12951-bib-0037] Tyner, S. D. , Venkatachalam, S. , Choi, J. , Jones, S. , Ghebranious, N. , Igelmann, H. , … Donehower, L. A. (2002). p53 mutant mice that display early ageing‐associated phenotypes. Nature, 415, 45–53. 10.1038/415045a 11780111

[acel12951-bib-0038] Veldurthy, V. , Wei, R. , Oz, L. , Dhawan, P. , Jeon, Y. H. , & Christakos, S. (2016). Vitamin D, calcium homeostasis and aging. Bone Research, 4, 16041 10.1038/boneres.2016.41 27790378PMC5068478

[acel12951-bib-0039] Zhang, H. , Davies, K. J. , & Forman, H. J. (2015). Oxidative stress response and Nrf2 signaling in aging. Free Radical Biology & Medicine, 88, 314–336. 10.1016/j.freeradbiomed.2015.05.036 26066302PMC4628850

[acel12951-bib-0040] Zhou, X. , Dai, X. , Wu, X. , Ji, J. , Karaplis, A. , Goltzman, D. , … Miao, D. (2016). Overexpression of Bmi1 in lymphocytes stimulates skeletogenesis by improving the osteogenic microenvironment. Scientific Reports, 6, 29171 10.1038/srep29171 27373231PMC4931581

[acel12951-bib-0041] Zittermann, A. , Gummert, J. F. , & Borgermann, J. (2009). Vitamin D deficiency and mortality. Current Opinion in Clinical Nutrition and Metabolic Care, 12, 634–639. 10.1097/MCO.0b013e3283310767 19710612

